# Rapid and Blind Watermarking Approach of the 3D Objects Using QR Code Images for Securing Copyright

**DOI:** 10.1155/2021/2236866

**Published:** 2021-11-16

**Authors:** Hanan S. Al-Saadi, Ahmed Elhadad, A. Ghareeb

**Affiliations:** ^1^Department of Mathematics, Faculty of Applied Sciences, Umm Al-Qura University, Makkah, Saudi Arabia; ^2^Computer Science and Information Department, College of Science and Arts, Jouf University, Sakakah, Saudi Arabia; ^3^Department of Computer Science, Faculty of Computers and Information, South Valley University, Qena, Egypt; ^4^Department of Mathematics, Faculty of Science, Al-Baha University, Al-Bahah, Saudi Arabia; ^5^Department of Mathematics, Faculty of Science, South Valley University, Qena, Egypt

## Abstract

Watermarking techniques in a wide range of digital media was utilized as a host cover to hide or embed a piece of information message in such a way that it is invisible to a human observer. This study aims to develop an enhanced rapid and blind method for producing a watermarked 3D object using QR code images with high imperceptibility and transparency. The proposed method is based on the spatial domain, and it starts with converting the 3D object triangles from the three-dimensional Cartesian coordinate system to the two-dimensional coordinates domain using the corresponding transformation matrix. Then, it applies a direct modification on the third vertex point of each triangle. Each triangle's coordinates in the 3D object can be used to embed one pixel from the QR code image. In the extraction process, the QR code pixels can be successfully extracted without the need for the original image. The imperceptibly and the transparency performances of the proposed watermarking algorithm were evaluated using Euclidean distance, Manhattan distance, cosine distance, and the correlation distance values. The proposed method was tested under various filtering attacks, such as rotation, scaling, and translation. The proposed watermarking method improved the robustness and visibility of extracting the QR code image. The results reveal that the proposed watermarking method yields watermarked 3D objects with excellent execution time, imperceptibility, and robustness to common filtering attacks.

## 1. Introduction

Digital watermarking has been proven effective for protecting digital media. It has recently gained considerable research interest. The watermarking process aims to embed secret data such that the resulting object is not greatly distorted. Also, the embedded watermark bits should resist malicious attacks to protect and/or verify the object ownership. Although the 3D objects are widely available and important, there are a few existing watermarking techniques. Therefore, the copyright of the 3D object needs more requesting to push research towards developing protection techniques. The various watermarking methods for 3D objects can be classified according to the embedding domains such as the spatial domain [1–3], the spectral domain [4, 5], and the transform domain [6, 7].

A mesh of a 3D object is a collection of polygonal facets that can be entirely described by two kinds of information: the geometry information describes the 3D positions (coordinates) of all its vertices, while the topology information provides the adjacency relations between the different elements [8, 9]. Considering these two attributes, watermark information can be added by modifying either of them [10]. Hence, they are usually called embedding primitives. Upon embedding, the quantity of the primitive is modified, typically by a very small amount, so that the watermarked model can still be used normally in any of its intended applications. Moreover, the watermark bits can be any stream of data to identify the owner while the Quick Response code (QR code) image stores data efficiently and has strong error correction capability [11, 12].

For document protection, in [13], Arkah et al. presented a color document watermarking technique based on embedding a QR code image into a document. The proposed method gets the document signature and information about the embedding and generates multi-QR codes to watermark the color document. The main contribution of the implemented prototype is to protect the color document against alteration and tampering. Moreover, in [14], Cardamone et al. proposed a nonblind watermarking method of documents for digital rights protection. The proposed method is using the QR code image that contains a signed ID of the user, and then it embeds the QR code image into the third level of the approximation coefficients from the discrete wavelet transform. On the other hand, in [15], Peng et al. generated a 3D QR code which is computed from their 2D counterpart. The 3D QR code has a special structure and is designed to be embedded in 3D shapes. The resultant QR code is 3D printable structures on any curved surface using homogeneous material.

In [16], Rosales-Roldan et al. presented three-color image watermarking techniques based on the singular value decomposition (SVD), discrete wavelet transform (DWT), and discrete cosine transform (DCT) which are used in the QR code image for authentication. The proposed methods apply Arnold permutation into the QR code image to prove the security. Thus, the proposed method uses the transformed luminance channel (Y) of the Y_C_b_C_r color space to embed the QR code image using the Quantization Index Modulation (QIM). In the same context, in [17], Patvardhan et al. presented a color image watermarking method that employs a combination between the discrete wavelet transform (DWT) and the singular value decomposition (SVD) for embedding the QR code image in a Y_C_b_C_r color space. The advantages of the proposed method are resistance to common attacks and providing good imperceptibility. Furthermore, in [18], Ran presented a QR code watermarking technique based on embedding the QR code itself in the spatial domain. The proposed method uses MD5 encryption and the logistic chaotic mapping algorithms to directly embed the watermark information into the original QR code image.

In [19], Chow et al. proposed a watermarking method for digital images using the QR code images and based on the discrete wavelet transform (DWT) and the discrete cosine transform (DCT). The proposed method decomposed the cover image using the discrete wavelet transform after it applied the discrete cosine transform on each block of the cover image. The QR code image was transformed using Arnold transform to increase security. Then two pseudorandom number sequences are generated to embed the QR code information in the DCT block of the cover image. The main idea of the proposed watermarking method benefits from the QR code structure that is inherent in the error correction to improve the robustness of the watermarking against attacks. Based on the discrete wavelet transform, in [20], Abdul et al. proposed a blind watermarking technique for images using the QR code.

In this paper, we are developing an enhanced rapid and blind method for producing a watermarked 3D object using QR code images with high imperceptibility and transparency. This paper is organized as follows.  Section 2 discusses materials and methods used for the 3D object watermarking method and related procedures. The proposed watermarking method is described in Section 3.  Section 4 presents the analysis and discussion of the experimental results. Finally, conclusions are summarized in Section 5.

## 2. Materials and Methods

This study aims to watermark the 3D object using a QR code to identify ownership rights of that original 3D object. The proposed method converts the 3D object vertices of the triangle from 3D coordinates to 2D coordinates by using the corresponding transformation matrix. Then, the watermarking step will be applied using the 2D coordinates of the triangle vertices and the QR code image pixel. The objective of digital watermarking can be summarized as embedding information into the “cover media” in such a way that the watermarked “Stego media” is perceptually indistinguishable from the original one. Furthermore, a good watermarking algorithm should be robust to removal or modification trials. This is of great importance especially if the watermark will be used to authenticate the source. Another critical issue with watermarking is how secure it is; in other words, how hard it is to decode the hidden information by an unauthorized user even if the watermarking technique is known.

### 2.1. The QR Code

The Quick Response code is always abbreviated to QR code which is a barcode that is readable by an imaging device such as a camera and smartphone. The QR code system was originally invented and designed in 1994 by the Japanese company Denso Wave and it was registered as a trademark of the same company [21, 22]. Simply, The QR code is a matrix code of two-dimensional barcodes and consists of black squares arranged in a square grid on a white background. Unlike the one-dimensional barcodes that were designed to be scanned by a narrow beam of light, the QR code is scanned by a digital image sensor and then digitally analyzed by a programmed processor. The QR code includes three main distinct squares at the corners to set up the image size normalization, orientation, and angle of viewing. Moreover, the small dots throughout the QR code are then converted to binary numbers and validated with the Reed–Solomon error-correcting algorithm [23] which are encoded as bytes of 8 bits. In practice, QR codes often contain data for a locator, identifier, or tracker that points to a standard URL for a website or application. A QR code uses four standardized encoding modes (numeric: Max. 7,089 characters, alphanumeric: Max. 4,296 characters, byte/binary: Max. 2,953 characters, and kanji: Max. 1,817 characters) to store the amount of data efficiently; extensions may also be used [23].

In this paper, the QR code generator is based on the ZXing (zebra crossing) library [24–26]. The QR code generator is software that creates data into a QR code image using the format information of two things: the error correction level and the mask pattern used for the symbol. The mask patterns are specified on a grid that is repeated as necessary to cover the whole symbol and protected from errors with a Bose–Chaudhuri–Hocquenghem (BCH) code and a couple of complete copies are included in each QR pattern. Hence, ZXing is an open-source library project implemented in Java, with ports to other languages which supports generating and decoding of multiformat 1D/2D barcode image processing such as QR code and Data Matrix within images and all files can be imported on the fly from a maven repository or can be downloaded via a command.  Figure 1 shows the generated four QR codes of size 69×69 which are used as an embedded image within the 3D objects.

### 2.2. Comparison Methods

In this study, the imperceptibility and the transparency performance analysis of the proposed watermarking method were evaluated between the original 3D object *u* and the watermarked object *v* by four different comparison methods. These include Euclidean distance, Manhattan distance, cosine distance, and the correlation distance. The Euclidean distance or Euclidean metric is the length measurement of a segment connecting between the two points in either the plane or 3-dimensional space in Euclidean space [27]. Therefore, it is the most obvious way of representing the differences between points in two 3D objects. It is given as the following equation:

(1) $$\begin{array}{c} \text{Euclidean dist}\left(u,v\right)=\sqrt{{\left|u_{x}-v_{x}\right|}^{2}+{\left|u_{y}-v_{y}\right|}^{2}+{\left|u_{z}-v_{z}\right|}^{2}}, \end{array}$$

where *u*_*x*_, *u*_*y*_, and *u*_*z*_ are the Cartesian coordinates of the original 3D object *u*. *v*_*x*_, *v*_*y*_, and *v*_*z*_ are the Cartesian coordinates of the watermarked object *v*.

The Manhattan distance, also known as the taxicab metric, is the sum of the absolute differences of Cartesian coordinates between two points [28]. This is known as taxicab distance because the shortest path that the car could take between two intersections has the same distance in taxicab geometry. The Manhattan distance is given as follows:

(2) $$\begin{array}{c} \text{Manhattan dist}\left(u,v\right)=\left|u_{x}-v_{x}\right|\;+\left|u_{y}-v_{y}\right|+\left|u_{z}-v_{z}\right|, \end{array}$$

where *u*_*x*_, *u*_*y*_, and *u*_*z*_ are the Cartesian coordinates of the original 3D object *u*. *v*_*x*_, *v*_*y*_, and *v*_*z*_ are the Cartesian coordinates of the watermarked object *v*.

Mathematically, the Cosine distance is a metric used to measure the cosine of the angle between the two 3D objects of an inner product space which is projected in a multidimensional space [29]. Thus, it is a judgment of orientation and not magnitude and determines whether the two objects are pointing in roughly the same direction which is given as follows:

(3) $$\begin{array}{c} \text{Cosine dist}\left(u,v\right)=1-\frac{u_{x}v_{x}+u_{y}v_{y}+u_{z}v_{z}}{\sqrt{{\left|u_{x}\right|}^{2}+{\left|u_{y}\right|}^{2}+{\left|u_{z}\right|}^{2}}\sqrt{{\left|v_{x}\right|}^{2}+{\left|v_{y}\right|}^{2}+{\left|v_{z}\right|}^{2}}}, \end{array}$$

where *u*_*x*_, *u*_*y*_, and *u*_*z*_ are the Cartesian coordinates of the original 3D object *u*. *v*_*x*_, *v*_*y*_, and *v*_*z*_ are the Cartesian coordinates of the watermarked object *v*.

The correlation distance is a statistic that measures the dependence between two 3D objects related to each other which is given as follows [30]:

(4) $$\begin{array}{c} \text{correlation dist}\left(u,v\right)=1-\frac{\left(1/3\left(-u_{x}-u_{y}-u_{z}\right)+u_{x}\right)\left(1/3\left(-v_{x}-v_{y}-v_{z}\right)+v_{x}\right)+\left(1/3\left(-u_{x}-u_{y}-u_{z}\right)+u_{y}\right)\left(1/3\left(-v_{x}-v_{y}-v_{z}\right)+v_{y}\right)+\left(1/3\left(-u_{x}-u_{y}-u_{z}\right)+u_{z}\right)\left(1/3\left(-v_{x}-v_{y}-v_{z}\right)+v_{z}\right)}{\sqrt{{\left|u_{x}+1/3\left(-u_{x}-u_{y}-u_{z}\right)\right|}^{2}+{\left|u_{y}+1/3\left(-u_{x}-u_{y}-u_{z}\right)\right|}^{2}+{\left|1/3\left(-u_{x}-u_{y}-u_{z}\right)+u_{z}\right|}^{2}}\sqrt{{\left|v_{x}+1/3\left(-v_{x}-v_{y}-v_{z}\right)\right|}^{2}+{\left|v_{y}+1/3\left(-v_{x}-v_{y}-v_{z}\right)\right|}^{2}+{\left|1/3\left(-v_{x}-v_{y}-v_{z}\right)+v_{z}\right|}^{2}}}, \end{array}$$

where *u*_*x*_, *u*_*y*_, and *u*_*z*_ are the Cartesian coordinates of the original 3D object *u*. *v*_*x*_, *v*_*y*_, and *v*_*z*_ are the Cartesian coordinates of the watermarked object *v*.

### 2.3. Converting 3D Coordinates to 2D Coordinates

Let us consider the basic representation of triangle vertices *A*,  *B*, and *C* in the 3D object coordinate system. So, there is a plane P defined with three points *A*(*xa*, *ya*, *za*),  *B*(*xb*, *yb*, *zb*), and *C*(*xc*, *yc*, *zc*) in the three-dimensional Cartesian coordinate system. Thus, for transforming the 3D coordinates to 2D coordinates and later restore coordinates using the transformation matrix, the first step is to set the A as the origin point of the coordinate system. The next step is to produce a new vector called *localz* that is perpendicular to both AB and AC using the cross product. Then, calculate *localx* which is the line segment that begins at the origin and ends at B. *localy* is the cross product between *localz* and *localx*. Finally, Figure 2 shows a piece of MATLAB source code to produce the transformation matrix.

Based on the above, the main contributions of this paper are as follows: (1) we introduce a 3D object watermarking method that hides a QR code image into the 3D object vertices; (2) we propose a blind extraction based on the reverse steps of the embedding process to recover the QR code image; (3) we brought evidence that the proposed watermarking method performed across the different 3D objects ensures a minimum shape distortion; (4) we present comprehensive experimentation examining the performance of our method and comparing it with other methods.

## 3. The Proposed Method

Assume that the 3D object information is stored in an STL file. This format describes only the surface geometry of a three-dimensional object without any representation of color, texture, or other common model attributes. So, the mathematical representation of the 3D object vertices is defined as *Obj*⊆ℝ^3^. In this study, Figure 3 illustrates a general model overview for the proposed method to watermark the 3D object using a QR code image. Each three vertices' coordinate in the *Obj* will be used to embed one-pixel value from the QR code image. The proposed method starts with converting the *Obj* triangles from the three-dimensional Cartesian coordinate system to the two-dimensional coordinates domain using the corresponding transformation matrix as mentioned in Section 2. Then, the watermarking process will be applied using the 2D coordinates of the vertices, QR code image, and a secret key. The watermarked 3D object will be constructed by the inverse of the modified *Obj* triangles to 3D coordinates.

### 3.1. The Watermarking Procedure

In this step, the watermarking process mainly focuses on embedding the QR code image into the 3D object. The proposed method applies a direct modification on the third vertex point of the *Obj* triangle in the 2D coordinates. Hence, let us assume that the three vertices of the current triangle in the 2D coordinates are *A*(0,  0), *B*(*x*,  0), and *C*(*x*,  *y*). There is a point *D*(*x*,  0) located on AB which is the projection of the Point C on AB. In this paper, the proposed embedding method calculates the point *D*'(*x*+Δ,  0) according to the current QR code image pixel to be using the following equation:

(5) $$\begin{array}{c} \text{distA}D^{\prime }=\;\frac{\text{distAB}}{\beta -1}\left(\frac{1}{255}\text{QRcode}+i\right)\;,\;\frac{i}{\beta -1}\text{distAB}\leq \text{distAD }\leq \;\frac{i+1}{\beta -1}\text{distAB},\;i=0,\;1,\;2,\;3,\;\cdots ,\;\beta -2, \end{array}$$

where distAB, distAD, and distA*D*′ are the Euclidean distance between *A*, *B*, and *D*′*QRcode* refers to the current pixel of the QR code image. An additional parameter *β* will be used for the embedding which indicates the number of intervals that will be used to divide the line AB distance. For security matter, the embedding process uses a Secret key to generate random permutation numbers such as [31, 32] which identified the current index of the Obj vertices. Moreover, to correctly retrieve the QR code image correctly and avoid the overflow problem, a preprocessing step is applied to the QR code image using a small integer value *α* as the following equation:

(6) $$\begin{array}{c} \text{QRcode}\left(\text{pixel}\right)=\left\{\begin{array}{cc} \alpha , & \text{pixel}=0,\\ 255-\alpha ,\; & \text{pixel}=255. \end{array}\right) \end{array}$$

Finally, the watermarked 3D object Obj' will be produced by restoring the 3D coordinates from the modified two-dimensional coordinates domain using the corresponding transformation matrix. The detailed steps of the watermarking process are listed in Algorithm 1.

### 3.2. The Extraction Procedure

In the extraction process, the steps carried out in the watermarking process are generally reversed to retrieve the QR code image using the secret key. Therefore, the extraction process starts with converting the 3D coordinates of the watermarked 3D object Obj' to 2D coordinates using the transformation matrix. Then, calculate the point *D*'(*x*',  0) on AB which is perpendicular from C'. In blind manner and using *β*, the QR code pixel will be calculated using the distance of AB and AD′ according to the following equation:

(7) $$\begin{array}{c} \text{QRcode}=\;255\left(\frac{\beta -1}{\text{distAB}}\text{distA}D^{\prime }-1\right)\;,\;\frac{i}{\beta -1}\text{distAB}\leq \text{distA}D^{\prime }\leq \;\frac{i+1}{\beta -1}\text{distAB,}\;i=0,\;1,\;2,\;3,\;\cdots ,\;\beta -2. \end{array}$$

Notice that the secret key is required to identify the index which is the current QR code pixel located. The detailed list of the extraction procedure steps is illustrated in Algorithm 2.

## 4. Results and Discussion

This section presents the performance and analysis results of the proposed watermarking and extraction algorithms using Egg [33], Bunny [34], Horse [34], and Cat Figurine [35] standard 3D objects.  Table 1 presents the detailed description of the number of vertices and maximum capacity in bytes for each 3D object and the corresponding image size in pixel of the used QR code and its decoded text in bytes as mentioned in Section 2.

### 4.1. Time Performance Results of the Proposed Algorithms

The proposed algorithms were implemented using Intel(R) Core (TM) i7-4700MQ CPU, 2.40 GHz processor with 8 GB of RAM. Moreover, the MATLAB version R2017b – 64 bits was used in coding the implementation. In addition, the parameters *α* and the secret key for the QR code image adjustment and the random permutation number generator were selected to be 5 and 1987, respectively.  Figure 4 records the execution time of the proposed watermarking and extraction process with *ß* values ranging from 100 to 1000 for each 3D object which was measured in terms of seconds. Clearly, the extraction execution time is less than the watermarking execution time for the same 3D object. Thus, the average time performance is 0.71, 0.69, 0.72, and 0.70 seconds for watermarking procedures Egg, Bunny, Horse, and Cat Figurine objects, respectively. The extraction process requires a little time of execution while it takes about 0.53, 0.52, 0.54, and 0.53 seconds for Egg, Bunny, Horse, and Cat Figurine models, respectively. Obviously, the parameter *ß* has a little impact on the time execution for the same embedded QR code image size where it is about 0.7 seconds and 0.5 seconds for embedding and extracting the 69 × 69 QR code image, respectively.

### 4.2. Imperceptibly and Transparency Performance Results

The imperceptibly and the transparency performances of the proposed watermarking algorithm were evaluated using Euclidean distance, Manhattan distance, cosine distance, and the correlation distance values whose details were explained in Section 2.  Figure 5 shows the obtained comparison results of the proposed method between the original 3D object and the watermarked 3D object using values of *ß* between 100 and 1000. The results show that higher values of *ß* offer a better visual quality of the watermarked 3D object. The resultant average values of the Euclidean distance for Egg, Bunny, Horse, and Cat Figurine models are 2.35, 0.81, 0.38, and 0.20, respectively. The average resultant Manhattan distances for Egg, Bunny, Horse, and Cat Figurine models are 175.34, 17.55, 4.11, and 1.39, respectively. The average resultant cosine distances for Egg, Bunny, Horse, and Cat Figurine models are 3.79E-06, 4.70296E-07, 8.84691E-08, and 4.63742E-08, respectively. The average resultant correlation distances for Egg, Bunny, Horse, and Cat Figurine models are 2.53E-05, 2.27E-06, 5.26E-07, and 1.73E-07, respectively.

Additionally, Figure 6 illustrates the corresponding resultant values of the Structural Similarity (SSIM) index of the extracted QR code image which is a perceptual metric that quantifies image quality degradation as perceived change in structural information [36] using the following equation:

(8) $$\begin{array}{c} \text{SSIM}\left(x,y\right)=\;\frac{\left(2\mu_{x}\mu_{y}+c_{1}\right)\left(2\sigma_{xy}+c_{2}\right)}{\left(\mu_{x}^{2}+\mu_{y}^{2}+c_{1}\right)\left(\sigma_{x}^{2}+\sigma_{y}^{2}+c_{2}\right)}, \end{array}$$

where µx and µy are the local means, and *σ*^2^_x_ and *σ*^2^_y_ are the variances of *x* and *y*. *σ*_xy_ is the cross-covariance for images *x*, *y*. *c*_1_ and *c*_2_ are variables to stabilize the division with a weak denominator. The illustrated results were provided using the values of *ß* between 100 and 1000. In fact, the results show that the various values of *ß* offer a small impact on the accuracy of the extracted QR code image. The minimum values of SSIM for Egg, Bunny, Horse, and Cat Figurine models are 0.999, 0.959, 0.947, and 0.966, respectively, and the maximum values of SSIM for Egg, Bunny, Horse, and Cat Figurine models are 0.999, 0.972, 0.974, and 0.972, respectively, while the average resultant SSIM for Egg, Bunny, Horse, and Cat Figurine models are 0.999, 0.966, 0.965, and 0.969, respectively. Furthermore, Figure 7 shows real samples of extracted QR code images from the 3D models using various values of *ß* where the extracted QR code images were decoded using ZXing library and the online tool Scan QR code and barcode from IMGonline.com.ua [37].

### 4.3. Robustness Performance Results

In this subsection, the robustness performance evaluation of the proposed watermarking method is investigated against the common 3D object filtering operations such as rotation, scaling, and translation. To prove the robustness of the proposed watermarking method, the Egg and Bunny watermarked 3D object when *β* = 500 were affected using the following attacks using open-source system MeshLab (v2016.12):

- Rotation (with rotation angle = 90°, 180°, and 270°)
- Scaling (with uniform scaling by 2, 3, and 4)
- Translation (with XYZ translation by -1, 0.5, and 1)

Table 2 illustrates the SSIM results of extracted QR code images after the previous types on the watermarked 3D object attacks. The extracted QR code image qualities are partially degraded after attacks; however it is remaining recognizable and decoded using ZXing library and the online tool Scan QR code and barcode from IMGonline.com.ua. Thus, the experimental result values prove that the proposed watermarking method maintains almost perfect retrieval of the QR code image and is robust against these attacks.

### 4.4. Comparison with Related Techniques

The main characteristics of the proposed method are compared with other existing methods to confirm its validity and efficiency. The comparative study is conducted in order to verify the used cover media, the watermark sequence, the embedding space, the domain, and the blindness extraction process between the proposed method and other methods.  Table 3 shows a comparison of the recorded details of the related methods. In [13, 14, 16, 17, 19], the presented methods were based on embedding the QR code into images based on various domains. On the other hand, in [1, 3] the presented methods were based on watermarking the 3D object using a different watermark sequence. Hence in this paper, the proposed 3D object watermarking method achieves the advantage characteristic of using the QR code as the embedding sequence into the 3D object.

## 5. Conclusions

This paper proposes a rapid watermarking method that embeds a QR code image in a 3D object based on the spatial domain. The proposed method starts with converting the 3D object triangles from the three-dimensional Cartesian coordinate system to the two-dimensional coordinates domain using the corresponding transformation matrix and then applying a direct modification on the third vertex point of each triangle. Each three vertices' coordinate in the 3D object can be used to embed one pixel from the QR code image by using the proposed watermarking algorithm. The extraction algorithm is totally blind based on the secret key and the reverse steps of the embedding process to recover the QR code image. The execution time of the proposed method to embed 225 bytes takes about 0.69 seconds; however, the extraction process takes 0.52 seconds for the same watermark bytes. The imperceptibly and the transparency performances of the proposed watermarking algorithm were evaluated using Euclidean distance, Manhattan distance, cosine distance, and the correlation distance values. The results show that higher values of *ß*, the division parameter, offer a better visual quality of the watermarked 3D object. The proposed method was tested under various filtering attacks, such as rotation, scaling, and translation. The proposed watermarking method improved the robustness and visibility of extracting the QR code image.

## Figures and Tables

**Figure 1:** QR code examples of size 69×69 and corresponding decoded text.

**Figure 2:** A piece of MATLAB source code to produce the transformation matrix.

**Figure 3:** A general model overview for the proposed watermarking and extraction method.

**Figure 4:** Time performance results of the watermarking and extraction algorithms.

**Figure 5:** The invisibility performance of the proposed watermarking method using Euclidean, Manhattan, cosine, and the correlation distances. (a) Euclidean distance. (b) Manhattan diatance. (c) Cosine distance. (d) Correlation distance.

**Figure 6:** The structural similarity results of the extracted QR code image.

**Figure 7:** Samples of extracted QR code images from (a) Egg, (b) Bunny, (c) Horse, and (d) Cat Figurine models.

**Algorithm 1:** Algorithm 1 The embedding procedure.

**Algorithm 2:** Algorithm 2 The extraction procedure.

**Table 1:** Description and capacity of the used 3D objects and QR code images.

Model	Vertices	QR code image size (pixels)	Secret text (bytes)	Max capacity (bytes)
Egg	40320	69 × 69	222	13440
Bunny	208353	69 × 69	225	69451
Horse	290898	69 × 69	216	96966
Cat Figurine	506910	69 × 69	232	168970

**Table 2:** Robustness results of the proposed watermarking method.

Test		Extracted QR code SSIM (Bunny)	Extracted QR code SSIM (Egg)
Rotation	Angle 90	0.9506	0.9993
	Angle 180	0.9437	0.9993
	Angle 270	0.9611	0.9993

Scaling	Uniform scaling by 2	0.9552	0.9993
	Uniform scaling by 3	0.9553	0.9993
	Uniform scaling by 4	0.9552	0.9993

Translation	XYZ translation by -1	0.9642	0.9993
	XYZ translation by 0.5	0.9642	0.9993
	XYZ translation by 1	0.9642	0.9993

**Table 3:** Main characteristics comparison of the proposed method with related methods.

Method	Cover media	Watermark sequence	Embedding color space	Domain	Is blind?
Chow et al. [19]	Grayscale image	QR code	Grayscale	DWT-DCT	Yes
Rosales-Roldan et al. [16]	Color image	QR code	YCbCr	SVD-DWT-DCT	Yes
Patvardhan et al. [17]	Color image	QR code	YCbCr	SVD-DWT	No
Arkah et al. [13]	Color document	QR code	RGB, gray	Spatial domain	Yes
Cardamone et al. [14]	Color document	QR code	RGB, gray	DWT	No
Ran [18]	QR code image	QR code	Binary image	Spatial domain	Yes
Jiang et al. [3]	3D object	Binary bits	Vertices	Spatial domain	Yes
Khalil et al. [1]	3D object	Gray image	Vertices	Spatial domain	Yes
The proposed	3D object	QR code	Vertices	Spatial domain	Yes

## Data Availability

The data that support the findings of this study are available from the corresponding author upon reasonable request.
